This article has been retracted.

# The role of seed appendage in improving the adaptation of a species in definite seasons: a case study of *Atriplex centralasiatica*

**DOI:** 10.1186/s12870-019-2090-6

**Published:** 2019-12-04

**Authors:** Zhaoren Wang, Yufei Zhao, Yuanyuan Zhang, Baoshan Zhao, Zhen’an Yang, Lijia Dong

**Affiliations:** 1 School of Life Sciences, Shaoxing University, Shaoxing, Zhejiang People’s Republic of China; 2 State Key Laboratory of Vegetation and Environmental Change, Institute of Botany, Chinese Academy of Sciences, Beijing, People’s Republic of China; 3 College of Life Science, China West Normal University, Nanchong, Sichuan, People’s Republic of China; 4 College of life science, Shanxi Normal University, Linfen, Shanxi People’s Republic of China; 5 University of Chinese Academy of Sciences, Beijing, People’s Republic of China

**Keywords:** *Atriplex centralasiatica*, Germination, Heteromorphism, Local adaptation, Seed appendages, Temperature and humidity

## Abstract

**Background:**

As a common accompanying dispersal structure, specialized seed appendages play a critical role in the successful germination and dispersal of many plants, and are regarded as an adaptation character for plants survival in diverse environments. However, little is known about how the appendages modulate the linkage between germination and environmental factors. Here, we tested the responses of germination to seasonal environmental signals (temperature and humidity) via seed appendages using *Atriplex centralasiatica*, which is widely distributed in salt marshlands with dry-cold winter in northern China. Three types of heteromorphic diaspores that differ in morphology of persistent bracteole and dormancy levels are produced in an individual plant of *A. centralasiatica*.

**Results:**

Except for the nondormant diaspore (type A, with a brown seed enclosed in a persistent bracteole), bracteoles regulated inner seed dormancy of the other two dormant diaspore types, i.e., type B (flat diaspore with a black inner seed) and type C (globular diaspore with a black inner seed). For types B and C, germination of bracteole-free seeds was higher than that of intact diaspores, and was limited severely when incubated in the bracteole-soaking solution. Dormancy was released at a low temperature (< 10 °C) and suitable humidity (5–15%) condition. Oppositely, high temperature and unfit humidity induced secondary dormancy via inhibitors released by bracteoles. Type C with deeper dormancy needed more stringent conditions for dormancy release and was easier for dormancy inducement than type B. The germination windows were broadened and the time needed for dormancy release decreased after the bracteole flushing for the two dormant types in the field condition.

**Conclusions:**

Bracteoles determine the germination adaptation by bridging seeds and environmental signals and promising seedlings establishment only in proper seasons, which may also restrict species geographical distribution and shift species distributing ranges under the global climate change scenarios.

## Background

Germination at an accurate time and space is important for plant local adaptation, ecological breadth and geographic distribution [1–3]. Germination time determines subsequent abiotic/biotic conditions in growth and reproduction period [4, 5], and acts as a selective force in the evolution of post-germination traits [1]. Many plants have elaborate checks on germination, which requires specific or even sequences of environmental conditions to release dormancy [2].

Seed dormancy is an adaptive trait that allows plants to optimize seedling establishments at proper time to ensure the completion of the plant life cycle within a suitable growing season [2, 6]. Two major types of dormancy mechanisms exist [7]. First, inherent dormancy resides within the embryo and/or the surrounding structures, such as the seed cotyledon, endosperm and seed coat, in which the balance among abscisic acid, gibberellins and ethylene controls seed dormancy and germination [8–11]. Second, seed appendage-imposed dormancy is conferred by the biomechanical mechanism [7, 12, 13]. Most studies in seed accompany structures focus on the mechanical inhibition in germination [13–15] and the benefits in seed dispersal [14, 15]. However, as ecologists noted, physiological dormancy is the most common type in the seven major dormancy classes [16, 17]. Little work has been done about the significance of biophysiological prevention, especially when linking with environmental conditions.

As Koller [18] and Baskin and Baskin [16] suggested, the germination ecology of a species cannot be understood unless intact natural dispersal units (seed or fruit, or with accessory parts) are considered. Embryo covering layers such as the seed coat and/or an indehiscent appendage creates mechanical resistance to seed germination [12, 13, 19] and shifts the duration of soil seedbank [13]. This information is a vital gap because the diversity of morphological and biomechanical inherent structures within seeds/fruits is the result of different strategies for successful dispersal and appropriate germination [20–23]. In addition, seed appendages also play as a pool of hormones for the regulation of seeds maturing process [24]. During the early developmental phase, many seed/fruit/diaspore are green and engaged in photosynthesis, where enzymes and hormones are produced [24]. Auxin and ABA in the pericarp of berries of grape (*Vitis vinifera* L.) controled the ripening time of berries [25]. Towards the end of the berry maturation phase, high levels of auxin were observed in the pericarp of high-SB (the ratio of seed weight to berry weight) berries.

In general, a variety of appendages are attached to the seeds of many species, and influence seed germination. For instance, the scarification of dispersal units could overcome the light limitation for germination of *Portulaca oleracea*, *Amaranthus deflexus* and *Oryza sativa* [16]. Also, removing the husks increased salinity tolerance of *O. sativa* seeds. Bracteoles on most species of *Atriplex* spp., pappi on *Taraxacum* spp., wings on *Ulmus* spp., *Acer* spp., *Salsola* spp. and arils on most species in *Celastraceae* spp. and *Marantaceae* spp. decreased seed germination owing to the presence of seed covering structures [16]. The inhibition effects of the covering structures are the results of mechanical restraint in water uptake, protrusion and gas exchange, and supply of inhibitors to the embryo [7, 12, 18, 26–28]. Special attentions are paid to the roles played by flavonoids, tannins, abscisic acid (ABA) and terpenes, particularly proanthocyanidins, in determining the physicochemical characteristics of the seed covering structures that influence seed dormancy, germination, and longevity in various species [7, 16]. For example, winged perianths of *Salsola komarovii* were found to make abscisic acid (ABA) [29], and many species in Eremophila produced water-soluble aromatic glycosides in the fruit walls that inhibited germination [30]. All the chemicals contained in appendages were shown to inhibit or delay germination, seeds would not achieve optimum germination unless the chemical inhibitors were leached by rainwater [27]. Furthermore, some seed appendages exhibit the release and then re-imposition of dormancy within the seed [15].

Interestingly, as Raviv et al. [24] reviewed, dead organs enclosing embryos (DOEEs), such as seed coats, pericarps and bract, were evolved not just for providing a physical protection for embryos or means for seed dispersal and germination but also as storage organs for active proteins, nutrients and metabolites for the purpose of germination, seedling establishments, nourishment and protection of germinating seeds from soil pathogens. The dead structures enclosing the fruits of several plant species contain various active enzymes involved in the hydrolysis process and detoxification of reactive oxygen species and therefore control seed germination. Hundreds of proteins were stored within DOEEs, which might further serve as an immediate nutritional supply for seedlings [31, 32]. Seedlings derived from intact diaspores had longer and more lateral roots than that derived from naked seeds [24, 32]. El-Keblawy et al. [33] assessed the roles of husks (dead lemma and palea) surrounding the grains of *Brachypodium hybridum* on germination behaviour and seedling growth and concluded that husks did not affect final germination or germination rate, but significantly enhanced seedling growth.

However, there are few systematic researches on the significance of appendages to species environmental adaptability. Most progresses address the function of seed appendages in anemochory, zoochory and hydrochory [15]. As the most direct sensor to environmental signals, seed appendages are paid little attention in their responses to environmental conditions. Furthermore, how do seed appendages modulate the linkage between germination of a species and environmental conditions over its distribution range in evolution? To demonstrate the significance of appendages on species fitness, we employed *Atriplex centralasiatica* Iljin to test the germination response of its seeds enclosed in bracteoles to temperature and rainfall, as its heteromorphic diaspores represent different dormancy types owing to different seed covering structures [34, 35].

*Atriplex centralasiatica*, a summer herbaceous halophyte in the family Amaranthaceae, is widely distributed in inland salt marshlands and coastlands in northern China. The inner seed is enclosed in the persistent bracteole for all dispersal units. *A. centralasiatica* distributing in the Otog Front Banner produces three types of diaspores (Fig. 1 a-c) in a plant or in a infructescence (Fig. 1d): the first type (Fig. 1a, left, further termed type A) is in a flat morph with a brown seed (Fig. 1a, right) enclosed in a bracteole slackly, the second type (Fig. 1b, left, further termed type B) is in a flat morph but with a black seed (Fig. 1b, right) enclosed in a bracteole firmly, and the third type (Fig. 1c, left, further termed type C) is in a globular morph with a black seed (Fig. 1c, right) enclosed in a bracteole firmly. Three kinds of heteromorphic diaspores differ in morphs and germination behaviours. Type A was kept in high germination potential until they were depleted in the following summer after maturity, while types B and C cycled between dormancy release (from maturing season in September to germinating season in March and April) and dormancy induction (the whole growing season from April to September) in the field [35, unpublished data]. The bracteole-free seeds germinate higher than intact diaspores [34]. To test the role of appendages in species fitness to environmental factors, we hypothesize that the seasonal fluctuation of temperature and precipitation governs the germination of inner seeds through bracteoles, and the appendage is the environmental condition sensor for seedling establishment. High temperature and humidity, simulated the condition of summer, can induce seeds into dormancy, while cold and dry condition occurring in winter can release seed dormancy, and the sensitive degree to hydrothermal condition was type A < type B < type C. Specifically, we ask the following questions: 1) what is the effects of bracteoles in heteromorphic diaspores on germination of inner seeds? 2) how does temperature and moisture regular germination through bracteoles? And 3) does the bracteole-modulated mechanism fit within the local adaptation of *A. centralasiatica* population?

**Fig. 1:** Three types of diaspores and their corresponding inner seeds from *Atriplex centralasiatica* (**a**-**c**), and a developing fascicled infructescence with heteromorphic diaspores (**d**). a, type A diaspore and seed; b, type B diaspore and seed; c, type C diaspore and seed

## Results

### Species distribution range and diaspore morphology

Most of *A. centralasiatica* populations distributed in northern China (Additional file 3: Figure S1), where the annual precipitation and the minimum monthly average temperature are less than 600 mm and 0 °C, respectively (Additional file 4: Figure S2a, b). The temperature and rainfall in the seed collection sites (i.e., Otog Front Banner) fluctuate with time, with a hot-humid summer and a cold-dry winter (Additional file 4: Figure S2c, d). Mass of diaspores was type A < type B < type C, while the mass of naked seeds was type A > type C > type B (Additional file 1: Table S1). Diaspore length, width and thickness of type B and C are large than type A (Additional file 1: Table S1a). The type A seed is larger in length and width, smaller in thickness and higher in water contend than the types B and C seeds (Additional file 1: Table S1b).

### The effect of bracteoles on germination and germination recovery from temperature- imposed dormancy

Three types of diaspores or seeds show significant differences in germination percentages. Over 80% of type A diaspores and bracteole-peeled seeds germinated in all treatments (Fig. 2 a, b). Fresh mature types B and C diaspores experienced < 5% and 0 germination, respectively (Fig. 2c, e). All nongerminated type A diaspores were dead, while all nongerminated types B and C were still viable after 30-day incubation. The bracteoles showed significant inhibition effects on germination of fresh and dormancy-break seeds (*P* < 0.001). Germination of dormancy-break types B and C diaspores, or seeds with their bracteoles were significantly inhibited by the bracteoles and decreased with incubation temperature (Fig. 2d, f), especially for type C (Fig. 2f). Nevertheless, the germination of bracteole-peeled seeds positively correlated with temperature. Unlike dormant diaspores (i.e., types B and C), type A diaspores had high germination under all temperature regimes and bracteole treatments (Fig. 2a).

**Fig. 2:** Effects of the diaspore type, bracteole and temperature on the germination (mean ± SE) of fresh and dormancy-break polymorphic diaspores and seeds of *Atriplex centralasiatica*. The left column represents germination of fresh, mature diaspores and seeds of type A (**a**), type B (**c**), and type C (**e**). The right column represents germination of dormancy-break diaspores or seeds of type A (**b**), type B (**d**), and type C (**f**). Diaspore, bracteoles attached to seeds; seed + bract, bracteoles removed from seeds but placed in the Petri dish with their seeds; seed, bracteoles removed from seeds

Recovery germination decreased with pretreatment temperature for dormancy-released diaspores and seeds with their bracteoles (Fig. 3), and it was lower for type C than for type B. No fresh seeds or diaspores regerminated in the recovery tests.

**Fig. 3:** The inhibition effect of bracteoles under three different temperature regimes on the subsequent recovery germination of type B (**a**) and type C (**b**) of *Atriplex centralasiatica*. Diaspore, bracteoles attached to seeds; seed + bracteole, bracteoles removed from seeds but placed in the Petri dish with seeds

### Seed imbibition tests

The temperature and bracteole had no significant effects on water imbibition of each type of seeds (Table 1), which means that the bracteoles and seed coats were water permeable at maturity. For two-type seeds, only type C seeds experienced more imbibition than diaspores at 20/30 °C. The mass of seeds increased > 50% for all treatments after water imbibition.

**Table 1:** The percentage of increased mass of seeds (i.e., naked seeds and seeds peeled from types B and C diaspores of *Atriplex centralasiatica*) after water imbibition

	Type B		Type C	
	5–15 °C	20/30 °C	5–15 °C	20/30 °C
Seed in diaspore	51.3 ± 4.9^Aa^	52.8 ± 2.6^Aa^	53.1 ± 0.5^Aa^	54.6 ± 0.7^Aa^
Naked Seed	55.7 ± 4.0^Aa^	52.6 ± 1.4^Aa^	59.0 ± 8.3^Aa^	59.1 ± 4.6^Aa^

Note, different capital letters indicate significant differences among different temperatures for the same type, and different lowercase letters indicate significant differences in imbibition between diaspores and seeds at the same temperature regime and seed type (mean ± SE, *n* = 4, *P* < 0.05, Duncan test)

### Leaching liquor

Germination of seeds incubating in bracteole leachates was significantly lower than incubating in distilled water (*P* < 0.001), particularly at 20/30 °C (Fig. 4). Furthermore, type C seeds were more sensitive to the leaching liquor, only 7 ± 2.5% (mean ± se, the same below) germinated at 20/30 °C in leachate, which was 97 ± 1.9% in distilled water.

**Fig. 4:** Effects of bracteole extracts and the temperature on germination of type B (**a**) and type C (**b**) seeds of *Atriplex centralasiatica*. Control, dormancy-break seeds incubated in distilled water. Leachate, dormancy-break seeds incubated in bracteole extracts

### Requirements of temperature and humidity for dormancy release

The limited window width of germination was reflected in the sensitivity of dormancy-released types B and C diaspores. Germination decreased rapidly as the temperature and humidity increased to 10 °C and 20%, respectively (Fig. 5). The magnitude of hydrothermal dormancy in diaspores recovering from cold stratification also reflected this changing environmental sensitivity. In general, dormancy increased to the highest level in August as soil temperature increased (unpublished data). Germination of types B and C diaspores decreased sharply in April and May, which implying monthly temperatures of 10.0 °C and 16.5 °C, respectively. Type C diaspores had narrower germination ridges than type B diaspores (Fig. 5). The hydrothermal limitation for diaspores dormancy break was depressed by extending the time of cold stratification.

**Fig. 5:** 3D plots of the germination percentage at different temperatures and humidities. Dormancy release at − 5, 0, 5, 10 °C and 0, 5%, 10, 15, 20% humidity conditions after a month cold stratification for type B (**a**) and type C (**c**) diaspores and two months cold stratification for type B (**b**) and type C (**d**) diaspores of *Atriplex centralasiatica*

### The effects of bracteole-leaching on seed germination and dormancy release

Diaspores of types B (Fig. 6a) and C (Fig. 6d) were covered with cavities after fillers were washed out by rainfall in the two-year placement in the field (type B: Fig. 6b; type C: Fig. 6e), or sharked for two hours on the shaker (type B: Fig. 6c; type C Fig. 6f). All the “filler” in the bracteoles of type C diaspores were flushed out, and the colour of type B bracteoles resembled type A after the rotation treatment.

**Fig. 6:** Diaspore morphologies of fresh type B (**a**), type B collected in the field after two-year placement on the soil (**b**), and water flushed type B (**c**), and fresh type C (**d**), type C collected in the field after two-year placement on the soil surface (**e**), and water flushed type C (**f**) of *Atriplex centralasiatica*

For diaspores and naked seeds of type B and type C, germination was significantly affected by cold stratification and temperature (Additional file 2: Table S2, *P* < 0.0001). Water flush (WF) only showed an obvious effect on type B diaspore germination. The fresh types B (Fig. 7a) and C (Fig. 7c) diaspores germinated less than 5% under the two conditions of no WF and WF. However, WF significantly improved the germination of dormancy-break types B (Fig. 7b) and C (Fig. 7d) diaspores (*P* < 0.001) and slowed the progression of temperature imbibition, especially at 10/20 °C and 15/25 °C. Germination windows were broadened widely for dormancy-break diaspores after fillers were washed out.

**Fig. 7:** The germination percentage of fresh diaspores of type B (**a**) and type C (**c**) of *Atriplex centralasiatica* and dormancy-released diaspores of type B (**b**) and type C (**d**) under different temperature regimes and soaking conditions

In the field experiments, bracteole-leaching broadened the germination window (Fig. 8a, c). Germination percentages increased significantly after leaching. Thorough flushing negated the inhibiting effects of high temperature and offset the difference between the two temperatures. The differences in germination percentages at 5/15 and 10/20 °C of type C diaspores were bigger than that of type B diaspores, unless flushed thoroughly. The germination index gradually increased with flushing time for type B diaspores, whereas a trend was not obvious for type C diaspores, except for flushing thoroughly (Fig. 8b, d). Salt content tests showed that the electrical conductivity of fresh mature diaspores was high but decreased sharply after a month of storage in the field (Additional file 5: Figure S3), which might have been leached out by rainfall.

**Fig. 8:** Germination trajectories of type B (**a**) and type C (**c**) diaspores and relative germination index of type B (**b**) and type C (**d**) of *Atriplex centralasiatica* at different incubation temperatures and flushing frequency after storage in field soil for 7 months

## Discussion

We found that the bracteoles of *A. centralasiatica* imposed a biochemical constraint on the germination of the encased seeds of the dormant diaspores. Germination patterns of *A. centralasiatica* polymorphic diaspores were modulated by bracteoles through identifying environmental signals (i.e., temperature and humidity). The seed appendages revised the germination requirements for environmental conditions upward, which limited germination windows and further, promised species establishment only in correct seasons.

### Inhibition via bracteoles

Bracteoles narrowed the germination of dormant seeds (i.e. type B and type C), but not the nondormant ones (i.e. type A). The primary dormancy of fresh mature seeds, such as type B and type C, might be set by maternal plants, aiming to prevent radical emergence during seed development until seed dry [36, 37]. However, it’s clear that the inhibition of germination after shedding is not set by the physiological dormancy (PD) of inner seeds and/or salt in the bracteoles. The reason is that even one time of rainfall could leach out salts that contained in the bracteoles. Furthermore, one-week cold stratification raised germination of naked seeds to over 90%, which is consistent with the findings from Li et al. [10] and Zhang et al. [35]. The restriction was imposed by their bracteoles and was shown in two processes, dormancy release and dormancy induce.

In the process of dormancy release**,** *A. centralasiatica* dormant diaspores lose bracteole-imposed dormancy over time in a process called after-ripening in the cold and dry winter after shedding. For the germination of inner seeds, their sensitivities to bracteoles decreased with temperature and moisture. The best opportunity for dormancy release is the time that unfavourable for seedling growth [16]. Bazin et al. [38] and Isabelle et al. [39] suggested that dormancy alleviation during after-ripening was associated with negative activation energies in distinct seed moisture conditions. In cool, temperate areas, the spring and early summer are the most favourable seasons for summer annuals germination, which provides the greatest probability for successful completion of species life history [2]. The dry and cold winter in Otog Front Banner offers suitable conditions for dormancy release. Dry conditions interrupted inhibitors transportation from bracteoles to seeds, and chilling enabled inner seeds to release PD [16]. The bracteoles postponed the process of dormancy release, and further reduced risks of germination after a transient favourable condition. Besides, bracteoles could confer significant ecological advantages by prolonging the dehydration process to allow seeds to retain sufficient water in germination, or decrease seed imbibition rates in the early stage to avoid germination in insufficient precipitation [40].

Bracteoles functioned a primarily express in dormancy inducement. Secondary dormancy was induced by high temperature and moisture conditions in late spring and summer. The leaching solution of bracteoles limited the germination of inner seeds. Rainwater and/or snowmelt act as mediums of inhibitors between inner seeds and exterior bracteoles. High temperature-activated inhibitors and further induced seeds into dormancy. Many structures that covering the embryo (i.e. endosperm, seed coats, indehiscent, fruit walls, palea/lemma, bracts, bracteoles and perianth) can restrict radicle emergence, especially for seeds with PD [16]. The chemicals in seed appendages such as flavonoids, tannins, terpenes, and semi-terpenes may inhibit the germination of inner seeds [7, 16]. In addition, bracteoles enhanced the inhibition of germination for fresh mature seeds, as no intact fresh diaspore germinated in any temperature regime. Without bracteoles covering on seeds, the non-deep physiological inhibition in the embryo could be effortlessly released by dry storage or cold stratification.

As the length of the favourable season for growth is projected to be shorten in temperate areas, such as arid and semi-arid deserts [41, 42], dormancy may be essential to prevent seeds from late germination. Dormancy of *A. centralasiatica* acted as a bet hedging, in which a fraction of diaspores remained in dormancy as a hedge against the risk of failure in completing regeneration [2, 43] and spreads offspring emergence over several possible germination windows [5]. Seasonal environmental conditions guide dormancy cycling and ensure seed germination in correct times [4, 27, 44–46]. Bracteoles drove the processes of dormancy release and dormancy induction and might be the bridge between the inner seed and external environmental signals. The increase in precipitation and temperature in late spring and early summer close germination windows of type B and type C diaspores. And bracteoles covering on seeds also keep fresh matured seeds in dormancy condition in the shedding season. In addition, the germplasm conservation mechanism guarantees the effective utilization of species germplasm resources in stressful conditions. It is noticeable that as predicted by previous studies [47–49], species germination decreased with temperature increase in the progress of global change, thereby, distribution ranges of *A. centralasiatica* may shift with the progress of global change according to this bracteole season-sensing system.

### Different adaptation strategies among polymorphic diaspores

Most plants only produce a single-type seed, and take monomorphism as their life-history strategy to cope with variable environments [16, 50]. However, three types of heteromorphic diaspores of *A. centralasiatica* functioned as a bet-hedging strategy to cope with the spatiotemporal variability of unpredictable habitats.

1. Fast-germinating diaspore type (Type A): it is a very fast germination type, according to the definition by Parsons [51]. Tiny restrictions of bracteoles on germination of type A diaspores were exhibited in all treatments. Type A diaspores commonly provide a competitive advantage in stress conditions. Tolerances to dry, heat and salinity in germination ensure rapid establishment of species in spring [10, 35]. Bracteoles would not affect germination of type A diaspore but may lengthen dispersal distance by wind, as they are much light and grow at the external layer of plant canopies. This is reverse to most species that seeds with a high degree of dormancy always combine with a high dispersal ability [14, 52, 53]. As observed in the field in Otog Front Banner in the arid/semi-arid area, are mainly established by type A diaspores. The dry autumn and winter may ensure type A diaspore storage until the beginning of the following rainy season. As nondormant seeds will necessarily predominate in subtropical environments [53]*,* we expect that, *A. centralasiatica* can colonize warm areas where plants developed from type A seeds are allowed to overwinter successfully.
2. Differences between types B and C diaspores: Globular type C diaspores might store more inhibitors in their bracteoles and be more sensitive to environmental signals than type B diaspores, which contributes to narrow emergence windows and keep a long-lived soil seedbank. Germination windows were open to June and May for types B and C diaspores in the field, respectively. Type C diaspores, which owning deeper dormancy and long-term seed banks, showed rapid responses to environmental changes and a sharp decrease in germination potential during the dormancy cycle in the field. Once air temperature and rainfall increased in late spring, type C diaspores were induced into secondary dormancy. This hypothesis is confirmed by a two-year soil seedbank experiment in the field where nearly no type C diaspore depleted but no type B diaspore remained after two years (unpublished data). We propose that these two types exploit the responsiveness of bracteoles to local abiotic cues in order to time the release of the bracteoles-imposed PD.

### Rainfall leaching

Flushing of bracteoles broadened germination capacity under limited conditions. Inhibitors in bracteoles were removed by precipitation in rainy seasons, thus gradually widening germination windows. Germination inhibitors being leached out by rainfall were corroborated by many other species with seed appendages [18, 27]. Dual roles are determined by the adaptive value of dormancy release via rainfall leaching. Fast dormancy release provides an opportunity for seedling establishment in a newly colonized habitat with adequate rainfall or abundant precipitation in an abnormal year. Alternatively, fast dormancy release also decreases the risk of seed mortality, which can be caused by predators, soil pathogens and intrinsic seed longevity [54].

Soaking appendages in water was reported as not promoting seed germination in many species [27]. However, this scenario is not contradictory to our results, since all their studies reviewing soaking used fresh mature diaspores. As noted in our study, leaching could not increase fresh diaspore germination but lifted the germination of dormancy-break diaspores. Debeaujon et al. [7] noted that complex interactions between the inner embryo and covering structures determine whether a seed will germinate. Dormant diaspores undergo a long process of after-ripening to enhance germination viability before emergence in the field. Dormant types B and C diaspores exhibit obvious differences in bracteole morphs. Bracteoles on globular type C hold more “fillers” than that in flat type B, and hold the “fillers” more firmly than type B by the covering cavities on the bracteole surface. The “fillers” constrained germination of seeds, and it was activated by soil temperature and moisture. Additionally, the inhibitors were leached to the soil by rain in the field, which may also avoid competitions with other species. As observed in the field, only *Peganum multisectum* could grow in the community that highly dominated by *A. centralasiatica*. Besides, as we tested, germination of *Suaeda salsa* and *Kalidium gracile,* two dominant species in Otog Front Banner, were restricted severely when incubated in the leaching solution of *A. centralasiatica* bracteoles. The inhibition effects may not only act on their encased seeds, but also on the germination of neighbor species, which needs to be further investigated.

## Conclusion

In this work, we found that germination of type B and type C diaspores of *A. centralasiatica* were modulated systematically by their bracteoles through sensing environmental signals (Fig. 9). High temperature and moisture activate inhibiting effects of bracteoles on the encased seeds, while the cold and dry conditions allow inner seeds to release dormancy. The bracteole-imposed dormancy disperses germination and seedling establishment over and beyond the actual growing season, and benefits *A. centralasiatica* for coping with such a fluctuating environmental condition in northern China. Rainfall leaching on bracteoles also optimized germination time by shifting dormancy pattern. According to the records of *A. centralasiatica* specimens, all the populations distributing in areas with average temperature below zero in January and average annual precipitation below 700 mm. We propose that the bracteoles with this biochemical mechanism contribute to the national distribution of this species in distinct environments. The subtle differences in the response of germination from polymorphic diaspores contribute to bet hedging adaptation for survival in seasonal habitats. Non-dormant diaspores (type A) and dormant diaspores (type B and type C) show obvious emergence differences and finally form the short-term and persistent seed banks. And furthermore, distribution ranges of *A. centralasiatica* may shift with the progress of global change according to this bracteole season-sensing system.

**Fig. 9:** Conceptual model of dormancy status and seedling regeneration of non-dormant diaspores (type A) and dormant diaspores (type B and type C) of *Atriplex centralasiatica*

## Methods

### Seed collection and site description

Freshly mature diaspores of *A. centralasiatica* were collected from natural populations growing on the edge of salt lakes in the Ordos Plateau of Inner Mongolia, northern China (38° 15′ 14′′ N, 107°28′ 52′′ E, 1314 m a.s.l.), on 20 Sep. 2016. Diaspores were air-dried under laboratory conditions for one week and then stored in a refrigerator at − 20 °C for subsequent experiments. We collected specimens from the populations and identified the species in accordance with “*Flora of China*” [55]. The specimens were stored in our laboratory, but not deposited as voucher specimens in herbarium. Pictures of the seedling, leaf, flower, stem, infructescence, individual and community of *A. centralasiatica* were shown in Additional file 6: Figure S4, which can be used for the verification of species identification.

The seed collection area has a typical continental, semi-arid climate with mean monthly temperatures from − 16.5 °C in January to 23.0 °C in July and annual precipitation of 254.3 mm. We downloaded and collected 375 reported *A. centralasiatica* specimens accounts providing complete collecting location information from the Chinese Virtual Herbarium (CVH, http://www.cvh.ac.cn/en), and mapped their location information on a map of China (QGIS 3.2.3). Cities where herbaria were collected were marked on the map except for those in Xinjiang, Gansu, Inner Mongolia and Qinghai-Tibet Plateau, where the herbaria were marked at county scales as counties in the above provinces were large enough and highly heterogeneous environments and landforms. Detailed habitats temperature and rainfall data across China from 1981 to 2010 were downloaded from the website of the China National Meteorological Data Service Center, China Meteorological Administration (CMDC, http://www.cma.gov.cn).

### The effects of bracteoles on germination and germination recovery from temperature- imposed dormancy

Germination of fresh and dormancy-break type B and type C diaspores was tested. Six months of dry storage under laboratory conditions and several-weeks of cold stratification (type B: 4-wk; type C: 8-wk) were used for the dormancy break, after which diaspores of types B and C germinated to 94.0 ± 2.6% and 92.0 ± 2.4%, respectively. Three types of treatments were employed to investigate the effects of bracteoles on the germination behaviours of heteromorphic diaspores: complete dispersal units, bracteole-peeled seeds with their detached bracteoles and bracteole-peeled seeds. Four replicates of twenty-five seeds of each treatment were set up in 5-cm-diameter plastic Petri dishes with two layers of Whatman No. 1 filter paper moistened with 3 ml distilled water. All the seeds and diaspores in the Petri dishes were sealed with parafilm and incubated for a photoperiod of 12 h (light)/12 h (darkness) at temperature regimes of 5/15, 10/20, 15/25, and 20/30 °C, representing approximately the mean daily minimum and maximum air temperatures in April and October, May and September, June and August and July, respectively. Germination (radical emergence) was recorded every 24 h until the 30th day or when all seeds or diaspores germinated. As Baskin and Baskin [16] suggested, germination tests had to be long enough to allow seeds sufficient time for germination, but it should not be so long that seeds can receive enough warm or cold stratification to break dormancy and thus promote germination. In addition, the ability of seeds to germinate within about 4-wk was one of criterion for dormancy classification [16]. For *A. centralasiatica*, most type A diaspores germinated within 7 days, while that for types B and C was from 5th to 25th days. In order to unify the incubating condition, we chose 30 days for all three types. All nongerminated type A diaspores were rotten after 30-day incubation.

To test the germination recovery from bracteole-imposed thermal dormancy, the ungerminated types B and C seeds or diaspores after 30d were transferred to Petri dishes with 3 ml distilled water after rinsing three times and then incubated for 30 d. Rinsed seeds and diaspores were cultured at 5/15 °C, which was the optimal temperature regimes for germination. As nearly all bracteole-peeled seeds germinated or decayed, these seeds did not undergo a recovery germination test. Recovery germination percentage (RG%) was determined as [a / (25 – b) × 100%, where a is the number of seeds germinated in new Petri dished after being transferred to distilled water, and b is the number of seeds germinated during the pre-treatment. All nongerminated diaspores were tested for viability using 0.4% TTC (Amresco, USA), and germination percentages were based on the number of viable diaspores.

### Seed imbibition tests

Dormancy-break type B and type C diaspores were used for the imbibition test. Diaspores in a similar size of type B (50 ± 3 mg) and type C (65 ± 3 mg) were randomly divided into two parts, with one part of the diaspores bracteoles peeled. Twenty-five dry seeds or diaspores of each type were weighted and then put into 5-cm-diameter Petri dishes with 3 ml distilled water. Four replicates of each treatment were placed in 5/15 and 20/30 °C for 48 h. As it is impossible to weigh a dry seed that enclosed in a bracteole, the mean mass of twenty-five bracteole-peeled dry seeds in the eight replicates was regarded as the initial weight of the seeds in the diaspores. The weight of soaked seeds or diaspores was measured after 48 h of water absorption. Each replicate of diaspores was weighed after the bracteoles were peeled. The water imbibition rate (Wr) of seeds was calculated as follows:

$$ {\mathrm{W}}_{\mathrm{r}}=\left[\left({\mathrm{W}}_{\mathrm{f}}-{\mathrm{W}}_{\mathrm{i}}\right)/{\mathrm{W}}_{\mathrm{i}}\right]\ast 100\left[16\right] $$

where W_f_ is the weight after 24 h, and W_i_ is the initial weight of seeds.

### Leaching liquor

Dormancy-break diaspores type B and type C were separated into seeds and bracteoles for the subsequent inhibition test. Eight Petri dishes of twenty-five type B and twenty-five type C bracteoles were soaked with 3 ml distilled water at 20/30 °C for 30 d. Then, all bracteoles were removed. Seeds were put into Petri dishes with their own leaching liquors and then incubated at 5/15 °C and 20/30 °C, which were the optimum temperature regimes for germination of diaspores and seeds, respectively. Incubation with distilled water served as a control. Germination was tested using the same procedure as those mentioned above.

### The effects of temperature and humidity on dormancy release

Diaspores of type B and type C were placed on two layers of filter paper and then placed into sealed metal boxes (20 cm length × 10 cm width × 10 cm depth) that were covered with washed, moist sand containing 0, 5, 10, 15 and 20% distilled water (e.g. the mean soil moisture is 10.6% in Otog Front Banner from November to the following March). The sealed metal boxes were kept in refrigerators at − 5 °C, 0, 5 °C and 10 °C in darkness. The temperature and moisture represent possible dormancy release conditions in the habitats and extreme conditions. Germination were tested in the same as those described in germination tests of fresh seeds and diaspores after 30 d and 60 d.

### The effects of bracteole leaching on dormancy release

To confirm that the bracteole inhibited inner seed dormancy release, fresh diaspores and bracteole-peeled seeds of type B and type C were used to investigate the effects of water flush (WF), dry storage, cold stratification and temperature treatments. Four replicates of two-hundred diaspores or seeds of each type that were placed into 1000-ml bottles with 200 ml distilled water were placed on the platform of a rock bed with a rotating speed of 60 r min^− 1^ for 2 h. As control subjects, diaspores or seeds in bottles without water were shaken on the same rock bed platform. Half of the rocked diaspores or seeds in the control and treatment groups were stored in closed envelope bags under laboratory conditions for six months. Following further treatment with 4-wk (type B) and 8-wk (type C) cold stratification for diaspores, 2-wk (type B) and 4-wk (type C) cold stratification for seeds, which were the optimal conditions for diaspores or seeds dormancy break. The control groups received the same storage time in a refrigerator at − 20 °C to maintain the primal state. Germination of the above-treated diaspores was tested under four temperature regimes (see the methods in ‘*The effects of bracteoles on the germination and recovery’* section).

To simulate the precipitation leaching effect on the inhibitors in bracteoles, we used the modified dynamic column elution method with simulated rainfall. Five sets of one-thousand type B and type C diaspores were placed under a 2 cm-aperture shower. The water was run at 0, 300, 600, 1500 and 3000 mm, which represented 0, 1, 2, 5, and 10 years rainfall flushing, respectively. Each set was packed in a closed cotton bag and placed in the field on September 30 (the shedding season) and returned on April 30 (emergence season). Germination was tested at 5/15 and 10/20 °C, which corresponded to the temperature regime of April and May, respectively (see the methods in ‘*The effects of bracteoles on the germination and recovery’* section). Germination rates (Gr) were also calculated as follows:

$$ \mathrm{Gr}={\sum}_{i=1}^{30}\frac{G_i}{D_i} $$

where *D*_*i*_ = days from start of the experiment to the *i*^*th*^ day observation. *G*_*i*_= number of diaspores germinated at the day *i*.

Non-flushed diaspores were collected on 30 Sep., 30 Oct. and 30 Mar. from the field for a salt content analysis of the bracteoles. Bracteoles peeled from type B and type C diaspores were dried for 48 h, ground into powder, and dissolved in 200 ml distilled water. The solid particles were filtered out of the suspension after 12 h, and then, electronic conductivity was tested (YSI-EXO1, Xylem, US).

### Data analyses

We compared germination proportions among treatments using the general linear model (GLM) tests, SAS Version 9.3 for windows (SAS Institute Inc., 2012). And data were arcsine transformed when necessary to meet assumptions of analysis of variance for normality, homogeneity of variance and multiple comparisons. Duncan’s test and paired two-tailed tests were performed for multiple comparisons to determine significant differences (*P* < 0.05) between individual treatments.

## Supplementary information

**Additional file 1: Table S1.** Mass, moisture content, and morphological characteristics types A, B and C diaspores and seeds of *Atriplex centralasiatica* (mean ± SE).

**Additional file 2: Table S2.** Three-way ANOVA analysis of variance for the germination of type B seed, type B diaspore, type C seed, and type C diaspore of *Atriplex centralasiatica* respectively.

**Additional file 3: Figure S1.** The main distribution area of *Atriplex centralasiatica* in China. Note: all the *Atriplex centralasiatica* populations are distributed in the temperate climate zones and Tibetan Plateau. Materials of diaspores were collected in Otog Front Banner. All 375 reported *A. centralasiatica* herbaria accounts from the Chinese Virtual Herbarium (CVH, http://www.cvh.ac.cn/en) and detailed habitats temperature and rainfall data across China from 1981 to 2010 were downloaded from the website of the China National Meteorological Data Service Center, China Meteorological Administration (CMDC, http://www.cma.gov.cn).

**Additional file 4: Figure S2.** Dynamics of mean monthly air temperature, precipitation in the whole distribution areas of *Atriplex centralasiatica* populations (a, b; mean, *n* = 30) and in Otog Front Banner where diaspores collected (c, d; mean, n = 30).

**Additional file 5: Figure S3.** The salinity of bracteoles peeled from type B and type C diaspores of *Atriplex centralasiatica* in September, October, and April next year.

**Additional file 6: Figure S4.** The phenotypic characteristic of *Atriplex centralasiatica* in the study site of Otog Front Banner in northern China.

## Data Availability

All data generated or analysed during this study are included in this published article.

## Abbreviations

Type A: type A diaspore, one kind of dispersal and germination unit produced by *Atriplex centralasiatica*, fan-shaped diaspores with brown seed enclosed in their bracteoles
Type B: type B diaspore, one kind of dispersal and germination unit produced by *Atriplex centralasiatica*, flat (fan-shaped) diaspores with black seed enclosed in their bracteoles
Type C: type C diaspore, one kind of dispersal and germination unit produced by *Atriplex centralasiatica*, globular diaspores with black seed enclosed in their bracteoles

## References

[1] Donohue K (2002). Germination timing influences naturalselection on life-history characters in *Arabidopsis thaliana*. Ecology.

[2] Donohue K, Rubio de casas R, Burghardt L, Kovach K, Willis CG (2010). Germination, postgermination adaptation, and species ecological ranges. Annu. Rev. Ecol. Syst..

[3] Kingsolver JG, Schemske DW (1991). Path analyses of selection. Trends Ecol Evol.

[4] Adondakis S, Venable DL (2004). Dormancy and germination in a guild of sonoran desert annuals. Ecology.

[5] Burghardt LT, Edwards BR, Donohue K (2016). Multiple paths to similar germination behavior in *Arabidopsis thaliana*. New Phytol.

[6] Finch-Savage WE, Leubner-Metzger G (2006). Tansley review: seed dormancy and the control of germination. New Phytol.

[7] Debeaujon I, Lepiniec L, Pourcel L, Routaboul J-M, Bradford KJ, Nonogaki H, Hoboken NJ (2011). Seed coat development and dormancy. Seed Development, Dormancy and Germination.

[8] Finkelstein R, Reeves W, Ariizumi T, Steber C (2008). Molecular aspects of seed dormancy. Annu Rev Plant Biol.

[9] Cyrek M, Fedak H, Ciesielski A, Guo Y, Sliwa A, Brzezniak L, Krzyczmonik K, Pietras Z, Kaczanowski S, Liu F (2016). Seed dormancy in Arabidopsis is controlled by alternative polyadenylation of DOG1. Plant Physiol.

[10] Li W, Liu X, Hanada A, Khan MA (2011). Effect of cold stratification, scarification and hormones on germination of dimorphic seeds of *Atriplex centralasiatica* under saline conditions. Seed Sci Technol.

[11] Verma V, Ravindran P, Kumar PP (2016). Plant hormone-mediated regulation of stress responses. BMC Plant Biol.

[12] Sperber K, Steinbrecher T, Kai G, Scherer G, Clausing S, Wiegand N, Hourston JE, Kurre R, Leubnermetzger G, Mummenhoff K (2017). Fruit fracture biomechanics and the release of *Lepidium didymum* pericarp-imposed mechanical dormancy by fungi. Nat Commun.

[13] Lu J, Tan D, Baskin CC, Baskin JM (2017). Role of indehiscent pericarp in formation of soil seed bank in five cold desert Brassicaceae species. Plant Ecol.

[14] Arshad W, Sperber K, Steinbrecher T, Nichols B, Jansen VAA, Leubner-Metzger G, Mummenhoff K (2019). Dispersal biophysics and adaptive significance of dimorphic diaspores in the annual *Aethionema arabicum* (Brassicaceae). New Phytol.

[15] Cousens RD, Dytham C, Law R (2008). Dispersal in plants. A population perspective.

[16] Baskin CC, Baskin JM (2014). Seeds: ecology, biogeography, and evolution of dormancy and germination.

[17] Willis CG, Baskin CC, Baskin JM, Auld JR, Venable DL, Cavender-Bares J, Donohue K, Rubio de Casas R, Group NGW (2014). The evolution of seed dormancy: environmental cues, evolutionary hubs, and diversification of the seed plants. New Phytol.

[18] Koller D (1957). Germination-regulating mechanisms in some desert seeds, IV. *Atriplex dimorphostegia* Kar. Et Kir. Ecology.

[19] Ohadi S, Mashhadi HR, Tavakol-Afshari R (2011). Effects of storage and burial on germination responses of encapsulated and naked seeds of turnipweed (*Rapistrum rugosum*) to light. Weed Sci.

[20] Mandák B, Pyšek P (2001). Fruit dispersal and seed banks in *Atriplex sagittata*: the role of heterocarpy. J Ecol.

[21] Mandák B, Pyšek P (2001). The effects of light quality, nitrate concentration and presence of bracteoles on germination of different fruit types in the heterocarpous *Atriplex sagittata*. J Ecol.

[22] Larson-Johnson K (2016). Phylogenetic investigation of the complex evolutionary history of dispersal mode and diversification rates across living and fossil Fagales. New Phytol.

[23] Steinbrecher T, Leubner-Metzger G (2018). Tissue and cellular mechanics of seeds. Curr Opin Genet Dev.

[24] Raviv B, Godwin J, Granot G, Grafi G (2018). The dead can nurture: novel insights into the function of dead organs enclosing embryos. Int J Mol Sci.

[25] Gouthu S, Deluc LG (2015). Timing of ripening initiation in grape berries and its relationship to seed content and pericarp auxin levels. BMC Plant Biol.

[26] Cresswell EG, Grime JP (1981). Induction of a light requirement during seed development and its ecological consequences. Nature.

[27] Ungar IA, Khan MA (2001). Effect of bracteoles on seed germination and dispersal of two species of Atriplex. Ann Bot.

[28] Sharma S, Amritphale D (2008). Light environment in pre- and post-dehiscent fruits affects seed germination in *Calotropis procera*. Environ Exp Bot.

[29] Takeno K, Yamaguchi H (1991). Diversity in seed germination behavior in relation to heterocarpy in *Salsola komarovii* Iljin. The botanical magazine.

[30] Richmond GS, Chinnock RJ (1994). Seed-germination of the Australian desert shrub eramophila (Myoporaceae). Bot Rev.

[31] Raviv B, Aghajanyan L, Granot G, Makover V, Frenkel O, Gutterman Y, Grafi G (2017). The dead seed coat functions as a long-term storage for active hydrolytic enzymes. PLoS One.

[32] Remans T, Nacry P, Pervent M, Filleur S, Diatloff E, Mounier E, Tillard P, Forde BG, Gojon A (2006). The Arabidopsis NRT1.1 transporter participates in the signaling pathway triggering root colonization of nitrate-rich patches. *Proc. Natl. Acad. Sci*. USA.

[33] El-Keblawy A, Elgabra M, Mosa KA, Fakhry A, Soliman S (2019). Roles of hardened husks and membranes surrounding brachypodium hybridum grains on germination and seedling growth. Plants.

[34] Li W, An P, Liu X, Khan MA, Tsuji W, Tanaka K (2008). The effect of light, temperature and bracteoles on germination of polymorphic seeds of *Atriplex centralasiatica* Iljin under saline conditions. Seed Sci Technol.

[35] Zhang R, Wang Y, Baskin JM, Baskin CC, Luo K, Hu X (2016). Germination and persistence in soil of the dimorphic diaspores of *Atriplex centralasiatica*. Seed Sci Res.

[36] Galloway LF, Etterson JR (2007). Transgenerational plasticity is adaptive in the wild. Science.

[37] Donohue K (2009). Completing the cycle: maternal effects as the missing link in plant life histories. *Philos. Trans. R. Soc. Lond., Ser. B: Biol*. Sci..

[38] Bazin J, Batlla D, Dussert S, Elmaaroufbouteau H, Bailly C (2011). Role of relative humidity, temperature, and water status in dormancy alleviation of sunflower seeds during dry after-ripening. J Exp Bot.

[39] Isabelle BS, Juliette L, Christophe B (2016). Fluctuation of Arabidopsis seed dormancy with relative humidity and temperature during dry storage. J Exp Bot.

[40] Chacon P, Bustamante RO (2001). The effects of seed size and pericarp on seedling recruitment and biomass in *Cryptocarya alba* (Lauraceae) under two contrasting moisture regimes. Plant Ecol.

[41] Venable DL (2007). Bet hedging in a guild of desert annuals. Ecology.

[42] Gremer JR, Kimball S, Venable DL (2016). Within-and among-year germination in Sonoran Desert winter annuals: bet hedging and predictive germination in a variable environment. Ecol Lett.

[43] Gremer JR, Venable DL (2014). Bet hedging in desert winter annual plants: optimal germination strategies in a variable environment. Ecol Lett.

[44] Footitt S, Clay HA, Dent K, Finchsavage WE (2014). Environment sensing in spring-dispersed seeds of a winter annual Arabidopsis influences the regulation of dormancy to align germination potential with seasonal changes. New Phytol.

[45] Footitt S, Douterelosoler I, Clay H, Finchsavage WE (2011). Dormancy cycling in Arabidopsis seeds is controlled by seasonally distinct hormone-signaling pathways. Proc Natl Acad Sci U S A.

[46] Hawkins KK, Allen PS, Meyer SE (2017). Secondary dormancy induction and release in *Bromus tectorum* seeds: the role of temperature, water potential and hydrothermal time. Seed Sci Res.

[47] Hoyle GL, Venn SE, Steadman KJ, Good RB, Mcauliffe EJ, Williams ER, Nicotra AB (2013). Soil warming increases plant species richness but decreases germination from the alpine soil seed bank. Glob Chang Biol.

[48] Rosbakh S, Poschlod P (2015). Initial temperature of seed germination as related to species occurrence along a temperature gradient. Funct Ecol.

[49] Seal CE, Daws MI, Flores J, Ortega-Baes P, Galíndez G, León-Lobos P, Sandoval A, Ceroni SA, Ramírez BN, Dávila-Aranda P (2017). Thermal buffering capacity of the germination phenotype across the environmental envelope of the Cactaceae. Glob Chang Biol.

[50] Walck JL, Hidayati SN, Dixon KW, Thompson K, Poschlod P (2011). Climate change and plant regeneration from seed. Glob Chang Biol.

[51] Parsons RF (2012). Incidence and ecology of very fast germination. Seed Sci Res.

[52] Buoro M, Carlson SM (2014). Life-history syndromes: integrating dispersal through space and time. Ecol Lett.

[53] Rubio de Casas R, Willis CG, Pearse WD, Baskin CC, Baskin JM, Cavenderbares J (2017). Global biogeography of seed dormancy is determined by seasonality and seed size: a case study in the legumes. New Phytol.

[54] Dalling JW, Davis AS, Schutte BJ, Elizabeth AA (2011). Seed survival in soil: interacting effects of predation, dormancy and the soil microbial community. J Ecol.

[55] Zhu G, Mosyakin SL and Clemants SE. Chenopodiaceae, In Wu CY, Raven PH, and Hong DY [eds.], Flora of China. 5, 365. Science Press, Beijing, China and Missouri Botanical Garden Press, St. Louis, Missouri, USA. 2003.

